The article "Application of 18F-FDG PET/CT in Langerhans Cell Histiocytosis" was published in 2022. Journal: Contrast Media Mol Imaging.

# Application of ^18^F-FDG PET/CT in Langerhans Cell Histiocytosis

**DOI:** 10.1155/2022/8385332

**Published:** 2022-08-19

**Authors:** Fengxiang Liao, Zhehuang Luo, Zizhen Huang, Rong Xu, Wanling Qi, Mingyan Shao, Pinggui Lei, Bing Fan

**Affiliations:** ^1^Department of Nuclear Medicine, Jiangxi Provincial People's Hospital, The First Affiliated Hospital of Nanchang Medical College, Nanchang 330006, Jiangxi, China; ^2^Sterilization and Supply Center, Jiangxi Provincial People's Hospital, The First Affiliated Hospital of Nanchang Medical College, Nanchang 330006, Jiangxi, China; ^3^Department of Radiology, The Affiliated Hospital of Guizhou Medical University, Guiyang 550000, Guizhou, China; ^4^Department of Radiology, Jiangxi Provincial People's Hospital, The First Affiliated Hospital of Nanchang Medical College, Nanchang 330006, Jiangxi, China

## Abstract

**Purpose:**

This study aims to explore the application value of the ^18^F-FDG PET/CT imaging in diagnosing, staging, and typing Langerhans cell histiocytosis (LCH) via the morphological and metabolic analyses of the ^18^F-FDG PET/CT images.

**Methods:**

We retrospectively analyzed the ^18^F-FDG PET/CT images and clinical data of nineteen patients with LCH. The shape, size, density, distribution, and ^18^F-FDG uptake of all lesions were documented. In addition, the SUVmax of the lesions, liver, and blood pool was measured prior to calculating the lesion-to-liver and lesion-to-blood pool ratios.

**Results:**

Among the 19 analyzed patients, the positive rate of the PET/CT image was 94.7% (18/19), with 1 false negative (5.3%, 1/19) case occurring in the cutaneous LCH. Among the 76 lesions, 69 were FDG-avid lesions (69/76, 90.8%). Additionally, we observed no FDG uptake in 7 lesions (7/76, 9.2%). In contrast, 59 lesions (59/76, 77.6%) were abnormal on diagnostic CT scan, but 17 lesions (17/76, 22.4%) were undetected. The ^18^F-FDG PET/CT image revealed additional 6 lesions in the bone, 4 in the lymph node, 3 in the spleen, and 3 occult lesions, which CT scan did not detect. Additionally, there were 6 cases with single-system LCH. The remaining 13 cases were multisystem LCH. Our ^18^F-FDG PET/CT image analyses altered the typing of 4 LCH patients. In the case of all lesions, the mean SUVmax of the ^18^F-FDG-avid lesions was 5.4 ± 5.1 (range, 0.8∼26.2), and the mean lesion-to-liver SUVmax ratio was 3.1 ± 2.52 (range, 0.7∼11.9), and the mean lesion-to-blood pool SUVmax ratio was 4.6 ± 3.4 (range 0.7∼17.5).

**Conclusion:**

The ^18^F-FDG PET/CT image plays an essential role in LCH diagnosis, primary staging, and typing. It can accurately evaluate the distribution, range, and metabolic information of LCH, providing a vital imaging basis for the clinical evaluation of disease conditions, selection of treatment schemes, and determining patient prognosis.

The article "Application of 18F-FDG PET/CT in Langerhans Cell Histiocytosis" was published in 2022. Journal: Contrast Media Mol Imaging.

## 1. Introduction

Langerhans cell histiocytosis (LCH) is characterized by the abnormal proliferation of Langerhans cells within the monocyte-macrophage system. It has dual characteristics of inflammation and tumor. Due to unknown etiology, atypical clinical manifestations, multiple tissues or organ involvement, and variable imaging findings, LCH diagnosis is difficult to achieve [1, 2]. LCH involves a single system performance for single or multiple lesions, and it can simultaneously apply a myriad of tissues and organs. Hence, its corresponding clinical treatment regimen can differ vastly, and its prognosis can vary greatly. For example, a single lesion requires surgery, while multiple lesions or multi-systems infiltration requires comprehensive treatment. Thus, clinical treatment needs to determine the distribution and extent of the lesion, especially in the infiltration of specific high-risk organs, such as the spleen, liver, lung, hematopoietic system, and central nervous system (CNS).

Traditional imaging evaluation has several advantages, like showing bone deterioration on an X-ray. Computed tomography (CT) offers better benefits for lung disease, while magnetic resonance imaging (MRI) can clearly display soft tissue and central nervous system lesions. However, due to a lack of overall characteristics, traditional imaging evaluation cannot detect whole-body lesions, which may introduce particular diagnostic challenges like missed lesions, improper assessment of disease activity, and so on. ^18^F-fluorodeoxyglucose positron emission tomography-computed tomography (^18^F-FDG PET/CT scan) is a multimodal molecular imaging technique that integrates functional metabolic and anatomical images. It can simultaneously obtain information on glycometabolic activity and systemic anatomy of lesions in one scan, which is very helpful for evaluating multisystem diseases. Previous studies and clinical applications revealed that ^18^F-FDG PET/CT could significantly improve the diagnostic accuracy of LCH and assess the disease activity and prognosis [3–5]. However, thus far, there is limited research on the application value of ^18^F-FDG PET/CT in LCH diagnosis [6]. Most reported studies were individual cases or had small sample sizes, and the results were controversial [7, 8]. Therefore, the potential metabolic features of LCH and the potential utility of ^18^F-FDG PET/CT in this field are unknown.

In this study, we collected the clinical data and PET/CT images of nineteen LCH patients with different ages of onset and single- or multisystem involvement. We summarized the PET/CT image-based morphological and metabolic characteristics of LCH patients to improve the understanding and diagnosis of this disease.

The article "Application of 18F-FDG PET/CT in Langerhans Cell Histiocytosis" was published in 2022. Journal: Contrast Media Mol Imaging.

## 2. Data and Method

### 2.1. Patient Selection

This study was a retrospective analysis. Nineteen patients pathologically diagnosed with LCH, who underwent the ^18^F-FDG PET/CT scan between June 2013 and April 2021, were enrolled in this study. The recruited patients underwent 22 ^18^F-FDG PET/CT scans between June 2013 and April 2021. All patients underwent a baseline ^18^F-FDG PET/CT scan before any treatment, 3 of whom also underwent one posttreatment FDG PET/CT scan. In addition, nineteen CT scans were performed for diagnosis or primary staging purposes, and 21 for restaging or follow-up. Meanwhile, 12 MRIs were performed. All baseline CT scans and/or MRI was obtained within 1 month before the PET/CT examination, and the images were clear (Table 1).

### 2.2. The ^18^F-FDG PET/CT Imaging Method

The fasting blood glucose (<11.1 mmol/L) levels were measured in all patients more than 6 hours before imaging. Next, ^18^F-FDG was intravenously injected at a dose of 0.10∼0.14 mCi/kg. Patients were allowed to lie down and rest for about 40∼60 minutes before the CT scan. The scanning range was from the top of the skull to the middle of the thigh, with layer spacing and layer thickness of 3.75 mm. Lastly, PET images were recorded in the same range in the 3D model. The acquisition time was 3 min/bed, and 6∼8 beds were collected. Following the iterative reconstruction of the images, the whole-body 3D maximum intensity projection (MIP) maps and transverse, coronal, and sagittal images were obtained. The ^18^F-FDG production, synthesis, and inspection equipment were GE MINIstrance cyclotron, Tracerlab FX chemistry auto synthesizer, and discovery STE, respectively. The radiological purity of the radiopharmaceuticals was greater than 95%.

### 2.3. Evaluation Method

#### 2.3.1. Subjective Judgment

The morphology, size, density, and ^18^F-FDG uptake in various parts of the entire body, including the bone, liver, spleen, lymph node, and lung, were observed macroscopically. The ^18^F-FDG PET/CT and CT images were reviewed independently by 2 high-level attending physicians in nuclear medicine to determine the anatomical location, morphology, density, and size of lesions on CT images, as well as the ^18^F-FDG uptake and distribution on PET images. A more senior physician was consulted in cases where the diagnosis was inconsistent.

#### 2.3.2. Quantitative Analysis

Quantitative analysis was performed with the standard uptake value (SUV = local tissue radioactivity concentration (kBq/kg)/(injected dose (kBq)/body weight (kg)) of ^18^F-FDG. The hypermetabolic lesion portion on PET was outlined with a 10 mm circle to delineate the region of interest (ROI) and measure the lesion maximum standard uptake value (SUVmax) for each pathological uptake liver SUVmax, and blood pool SUVmax values [6]. Next, we calculated the lesion-to-liver SUVmax and lesion-to-blood pool SUVmax ratios. The maximum and minimum diameter of the lesion, splenic rib unit, and pituitary thickness were also measured, and the numbers were recorded on CT images.

The article "Application of 18F-FDG PET/CT in Langerhans Cell Histiocytosis" was published in 2022. Journal: Contrast Media Mol Imaging.

#### 2.3.3. Imaging Evaluation Criteria

PET positivity, representing enhanced metabolism, described a higher lesion ^18^F-FDG uptake than the liver. In this case, lesion SUVmax > liver SUVmax. Moreover, the FDG uptake of physiological, reactive, or other diseases was excluded due to clinical and other imaging. PET negative was defined as no significant FDG uptake or FDG uptake less than the liver SUVmax.

On CT imaging, the following were considered to represent positive lesions: abnormalities in morphology, structure, size, or density that physiologic or other diseases could not explain. This included bone destruction, a short diameter of the lymph nodes (greater than 10 mm), abnormal low-density lesions in the liver and lung, spleen with more than 5 intercostal spaces, and so on.

#### 2.3.4. Classification and Typing

According to the LCH phase III trial by the International Histiocyte Association, LCH was divided into ① single-system Langerhans cell histiocytosis (SS-LCH): one organ/system involvement (single or multiple lesions); ② multisystem Langerhans cell histiocytosis (MS-LCH): more than two organs/systems involvement. In addition, they were classified into high- and low-risk groups based on the presence or absence of “organ at risk” involvement—bone marrow, spleen, liver, and lungs [1, 9].

### 2.4. Statistical Analysis

SUVmax of the ROI was measured using SPSS 19.0 and is expressed as mean ± standard deviation, and the analysis was performed using a *t*-test. The positive rates of ^18^F-FDG PET/CT and CT images were compared using the *χ*^2^-test. Finally, *P* ≤ 0.05 was considered statistically significant.

## 3. Results

### 3.1. Patient Characteristics and Lesion Location

Among nineteen LCH patients, 7 were males, and 12 were females, between the ages of 0.5 to 66 years, with an average age of 24.3. In addition, 9 cases were older than 18 years (3 male and 6 female, mean age: 48.1 years old), 10 subjects were younger than 18 years (4 male and 6 female, mean age: 2.95 years old), and 5 cases were younger than 2 years (0 male and 5 female, mean age: 0.9 years old).

The article "Application of 18F-FDG PET/CT in Langerhans Cell Histiocytosis" was published in 2022. Journal: Contrast Media Mol Imaging.

A total of 76 lesions were pathologically or clinically identified in nineteen patients with LCH, and the location distribution is summarized in Table 2. Among the nineteen patients, the positive rate of PET/CT was 94.7% (18/19), which showed the presence of at least one hypermetabolic lesion consistent with LCH, and 1 false negative (5.3%, 1/19) case occurred in the cutaneous LCH.

Among the 76 lesions, 69 were FDG-avid lesions (69/76, 90.8%). Seven lesions (7/76, 9.2%) were found to have no FDG uptake, including 1 pituitary stalk lesion, 2 lung vesicles, 1 vertebral osteogenic lesion, 1 small round hypodense liver foci, and 1 abdominal lymph node lesion. Conversely, 59 lesions (59/76, 77.6%) were abnormal on diagnostic CT, but 17 lesions (17/76, 22.4%) appeared normal. The abnormal lesion locations were as follows: 1 skin lesion, 1 pituitary stalk lesion, 1 labia lesion, 1 auricle lesion, 3 spleen lesions, 4 lymph node lesions, 2 iliac lesions, 1 vertebra lesion, 1 femur lesion, 1 humerus lesion, and 1 temporal bone lesion, respectively (Table 3).

### 3.2. PET/CT Image Features

The ^18^F-FDG PET/CT images and metabolism of nineteen patients are shown in Tables 2 and 3. There were 14 LCH cases with bone infiltration (34 lesions). Among them, 28 lesions exhibited penetration or osteolytic bone destruction, most of which were combined with soft tissue mass. In addition, ^18^F-FDG uptake increased in 27 lesions with SUVmax of 2.6∼23.2. One vertebral lesion showed entophagocytic bone destruction without significant ^18^F-FDG uptake. One vertebral lesion showed patchy high-density shadow and osteogenic changes on CT but no significant ^18^F-FDG uptake. Similarly, 6 lesions showed normal bone morphology on CT (1 in the vertebral body, 1 in the humerus, 1 in the femur, 1 in the temporal bone, and 2 in the iliac bone). In addition, there were eleven LCH cases with lymph node infiltration (24 lesions). Among them, 20 lesions exhibited enlarged lymph nodes of varying degrees, with a short diameter of 10 mm∼36 mm; 4 lesions had lymph nodes with a short diameter of <10 mm; and 23 lesions showed increased ^18^F-FDG uptake with SUVmax of 2.5∼20.4.

Three LCH cases displayed lung infiltration. Among them, 1 primary case showed an extensive mass, nodular high-density shadow, and central necrosis in both lungs, with increased ^18^F-FDG uptake and SUVmax of 8.9∼10.2. Two multisystem LCH cases with lung infiltration included 1 case with strip consolidation in the upper lobe of the right lung, a slight increase in ^18^F-FDG metabolism, as well as a SUVmax of 4.3, and 1 case with extensive cystic low-density shadow in both lungs, as well as no significant ^18^F-FDG uptake (Figure 1).

The article "Application of 18F-FDG PET/CT in Langerhans Cell Histiocytosis" was published in 2022. Journal: Contrast Media Mol Imaging.

We also detected three multisystem LCH cases with liver infiltration. Among them, 1 case showed mild liver enlargement with diffused elevation in ^18^F-FDG uptake and SUVmax of 2.8; two cases showed multiple small round low-density shadows in the liver, including 1 case with increased ^18^F-FDG uptake as well as SUVmax of 4.6, and 1 case without significant ^18^F-FDG uptake. On CT, three multisystem LCH cases with spleen infiltration exhibited no substantial changes in form or size, with a dispersed elevation of ^18^F-FDG uptake and SUVmax of 2.6∼5.9 (see Figure 2). On CT, one LCH patient with thyroid infiltration had widespread goiter, with considerable increases in ^18^F-FDG absorption and a SUVmax of 9.6. On MRI, one LCH case with diabetes insipidus showed thickening of the pituitary stalk and decreased signal of the posterior pituitary, but no apparent abnormalities in ^18^F-FDG PET or CT. One LCH case with skin infiltration had only a skin rash, with no discernible abnormalities on ^18^F-FDG PET or CT. One LCH patient with auricle infiltration had a small nodular soft tissue density near the bilateral auricles, increased ^18^F-FDG uptake, and a SUVmax of 4.5. Finally, one LCH case had labia infiltration with only slightly thickened outer labia, increased ^18^F-FDG uptake, and a SUVmax of 8.6.

For all lesions, the mean SUVmax of the ^18^F-FDG-avid lesions was 5.4 ± 5.1 (range, 0.8∼26.2), and the mean lesion-to-liver SUVmax ratio was 3.1 ± 2.52 (range, 0.7∼11.9), and the mean lesion-to-blood pool SUVmax ratio was 4.6 ± 3.4 (range, 0.7∼17.5). For the 14 bone localizations of LCH, the average SUVmax was 6.7 ± 6.8 (range, 1.4∼26.2), and the average lesion-to-liver SUVmax ratio was 3.7 ± 2.8 (range, 1.7∼11.9). The average lesion-to-blood pool SUVmax ratio was 5.6 ± 4.5 (range, 1.2∼17.5). For the 11 lymph node localizations of LCH, the average SUVmax was 5.9 ± 4.3 (range, 1.8∼16.9), and the average lesion-to-liver SUVmax ratio was 3.4 ± 2.0 (range 0.9∼7.7). The average lesion-to-blood pool SUVmax ratio was 5.0 ± 3.0 (range, 1.5∼11.3). Patients with multisystem or multiple-site involvement of a single system did not exhibit significantly elevated baseline SUVmax values, lesion-to-liver SUVmax ratios, or lesion-to-blood pool SUVmax ratios compared to the single-site involvement patients.

### 3.3. Classification and Typing

The 6 cases of single-system LCH included 3 cases of single site and 3 cases of multiple sites. The single-site patients had eosinophilic granuloma (EG) involvement in the parietal, rib, and frontal bones. Patients had infiltration in the lung, bone, and skin at different places. One case of multisystem LCH was in the low-risk group, while 12 cases were in the high-risk group. The patient in the low-risk group had the presence of the cervical and mediastinal lymph nodes, the thyroid gland, auricle, and external labia. Among the twelve patients in the high-risk group, 4 experienced bone marrow and lymph node involvement, and these were the most prominent cases. Refer to Table 4 for the classification and typing of the nineteen LCH patients.

The article "Application of 18F-FDG PET/CT in Langerhans Cell Histiocytosis" was published in 2022. Journal: Contrast Media Mol Imaging.

## 4. Discussion

The LCH is a rare clonal disease originating from the bone marrow monocyte-macrophage system. The underlying mechanism involves CD1*α*+/CD207 + dendritic cells (DCS) proliferating out of control due to continuous immune stimulation. LCH is characterized by granulomatous lesions composed of clonal pathological tissue cells. Zinn et al. reported that LCH is more prevalent in children and males (M/F = 1.2∼1.4), with an annual incidence rate of 4∼8/million in children and 1∼2/million in adults, respectively [2]. However, in this study, the number of children (10/19) and adults (9/17) with LCH were almost the same. Moreover, the number of males (7/19) was significantly less than that of females (12/19) (M/F = 0.58). This discrepancy in data between our research and the presented article may be due to the gradual rise in adult LCH incidence. LCH can invade all tissues and organs of the body. Based on prior reports, the most common sites of LCH lesions are the bone (80%), skin (33%), pituitary (25%), liver (15%), spleen (15%), hematopoietic system (15%), lung (15%), lymph nodes (5∼10%), and CNS excluding pituitary (2∼4%) [10]. However, in this study, the most common sites were the bone (14/19), lymph nodes (11/19), lung (3/19), liver (3/19), spleen (3/19), auricle (2/19), thyroid, skin, pituitary, and outer labia (all 1/19). Compared to the earlier studies, our research found more lymph node involvement, less skin and nervous system (including pituitary) involvement, and no involvement of the salivary gland and digestive tract. This is likely because not all lymph node lesions were confirmed by pathology, and some skin and CNS involvement were missed owing to the negative result on ^18^F-FDG PET/CT.

Langerhans cells, lymphocytes, and eosinophils in LCH had high glucose affinity. Thus, LCH-driven lesions exhibited high glucose metabolic activity on ^18^F-FDG PET/CT imaging. Based on our results, PET/CT found more lesions than diagnostic CT in both the bone and lymph node lesions. PET/CT sometimes detected additional lesions with normal skeletal morphology on CT. In our study, 6 bone lesions, without bone destruction, were not detected by CT but were found in PET/CT due to increased ^18^F-FDG uptake. However, PET/CT is not as sensitive as CT in displaying osteogenic lesions. Relative to MRI, it was reported that PET alone is less susceptible to spinal lesions [11]. In the case of lymph node and spleen lesions, routine imaging examinations determine whether the lesions are abnormal or not, based on size. However, some lymph nodes (short diameter <10 mm) or normal-sized spleens may also be involved. The study discovered high uptake of ^18^F-FDG in 4 lymph nodes with a short diameter of <10 mm and 3 normal-sized spleens. Alternately, ^18^F-FDG PET/CT had a specific false positive rate in LCH diagnosis with lymph node infiltration. Sometimes, it was challenging to distinguish LCH from inflammatory hyperplasia. For example, 3 hypermetabolic cervical lymph node biopsies showed significant inflammation. Despite this, PET/CT can guide the clinical selection of reliable biopsy sites.

The article "Application of 18F-FDG PET/CT in Langerhans Cell Histiocytosis" was published in 2022. Journal: Contrast Media Mol Imaging.

In the case of lung lesions, ^18^F-FDG PET/CT is sometimes inferior to conventional diagnostic CT [12, 13], especially in examining pulmonary vesicles. Small nodules and interstitial changes often appear negative on ^18^F-FDG PET/CT. It may be related to the fact that the small nodules (less than 5 mm) and the thin capsule wall exceed the spatial resolution of PET/CT. A case of extensive cystic density lesion of both lungs failed to demonstrate ^18^F-FDG uptake. Therefore, diagnostic CT, exceptionally high-resolution CT (HRCT), must be conducted when lung involvement is suspected. It was previously reported that only 1 out of 4 LCH cases with lung infiltration showed high uptake of ^18^F-FDG [6]. Another study revealed that thyroid LCH could be mistaken for Hashimoto's thyroiditis and thyroid papillary carcinoma. In the case of multisystemic LCH, with suspected thyroid infiltration, it is recommended to puncture under ultrasound guidance to ensure a definite pathological diagnosis [14]. But, we made no such discovery in this study. Studies reported that ^18^F-FDG PET/CT is inferior to MRI when imaging the nervous system, including the pituitary [15]. A case of diabetes insipidus showed thickening of the pituitary stalk and decreasing posterior pituitary signal on MRI, but no abnormality was evident on PET/CT.

Additionally, LCH with skin infiltration in infants is often misdiagnosed as seborrheic dermatitis and refractory diaper dermatitis [16] due to the difficulty of detecting specific abnormalities on PET/CT. On the contrary, PET/CT helps detect certain hidden diseases. For example, lesions of the auricle and external labia were easily detected using PET/CT in this study. Some scholars [17] also revealed that PET and CT identified lesions missed on conventional imaging and helped decipher whether a lesion was active or inactive.

The article "Application of 18F-FDG PET/CT in Langerhans Cell Histiocytosis" was published in 2022. Journal: Contrast Media Mol Imaging.

The ^18^F-FDG-PET/CT imaging has several advantages, including integrating anatomical and functional metabolism information, creating a whole-body image in one scan, and comprehensively evaluating whole-body involvement. All these are beneficial to staging and typing, particularly the assessment of “dangerous organ” involvement. It is essential to confirm the type of LCH as early as possible, as the treatment and prognosis of a single LCH (SS-LCH) and multisystem of LCH (MS-LCH) are vastly different. SS-LCH with a single lesion is often treated via surgery, whereas SS-LCH with multi-lesions or MS-LCH is treated via a combination of radio- and chemotherapies. SS-LCH with multifocal bone lesions is rarely fatal but may relapse and lead to related sequelae [18]. It was reported that a BRAF mutation in MS-LCH regulates pluripotent hematopoietic primordial cells [19]. The PET/CT detected 11 additional lesions (11/76) in this study. Out of which 2 spleen and 2 lymph node infiltration changed the classification of 4 patients; 1 case was upgraded from SS-LCH with a single lesion to MS-LCH, and 3 cases were upgraded from SS-LCH with multiple lesions to MS-LCH.

Unfortunately, our work encountered certain limitations. Firstly, not all positive PET/CT lesions were confirmed via pathology, leading to the possibility of false positives. Secondly, our case sample population was relatively small and required further validation with a larger sample size and multi-center collaboration. Lastly, although 3 patients underwent PET/CT examination after treatment, this article did not analyze the value of PET/CT in the efficacy evaluation of LCH, and additional studies are warranted to validate our results.

## 5. Conclusion

In conclusion, ^18^F-FDG PET/CT imaging is critical for LCH diagnosis, initial staging, and typing. The PET/CT detects more lesions involving the LCH than diagnostic CT. As a result, we recommend PET/CT for the detection, staging, and typing of LCH, which will provide a critical imaging foundation for the clinical evaluation of disease conditions, treatment scheme selection, and prognosis of LCH patients.

## Figures and Tables

**Figure 1:** Female, 1 year old, MS-LCH (bone marrow + lung + lymph nodes). (a, b) Extensive cystic low-density shadow in both lungs without significant ^18^F-FDG uptake. (c) Enlarged lymph nodes in the anterior mediastinum increased ^18^F-FDG uptake and SUVmax of 5.7. (d, e) Penetrating bone destruction and local soft tissue density shadow in the left temporal bone and mandible increased ^18^F-FDG uptake and SUVmax of 6.4. (f) Bilateral cervical multiple enlarged lymph nodes on CT, with the larger one of 15 × 11mm, but without significant ^18^F-FDG uptake. LCH infiltration was excluded via pathology.

The article "Application of 18F-FDG PET/CT in Langerhans Cell Histiocytosis" was published in 2022. Journal: Contrast Media Mol Imaging.

**Figure 2:** Female, 35 years old, MS-LCH (lymph nodes + bone marrow + spleen). A1 was PET MIP; B1 was CT cross-section; C1, D1, E1, and F1 were PET/CT fusion, respectively. A1 showed multiple enlarged lymph nodes observed in the bilateral neck, pelvic cavity, and retroperitoneum, with increased FDG uptake and SUVmax of 8.7. B1 showed bone destruction at the frontal bone of the left side, with no significant increase in FDG uptake (C1); D1 showed no enlargement of the spleen but diffusely increased FDG uptake when SUVmax was 5.6. E1 showed increased thoracic bone density and slightly increased FDG uptake with SUVmax of 2.9. F1 showed increased focal FDG uptake in the left iliac crest with SUVmax of 5.3. PET/CT was performed after 8 cycles of chemotherapy. A2 was PET MIP; B2 was CT cross-section; and C2, D2, E2, and F2 were PET/CT fusion. A2 showed no abnormal increase in FDG uptake, B2 showed basic repair of the left frontal bone, D2 spleen metabolism reduced to normal, E2 high-density shadow became weak, and metabolism decreased, and F2 left iliac bone lesion metabolism dropped to normal.

**Table 1:** The population and categorization of imaging examination used in this study.

Variables	Imaging categorization	Frequency
Gender	Female	12
	Male	7

Age	Average age (range)	24.3 (0.5～66)
	Older than 18 years	9
	Younger than 18 years	10
	Younger than 2 years	5

Imaging examination	PET/CT scan	22
	PET/CT scan before treatment	19
	PET/CT scan after treatment	3
	Diagnostic CT scan	40
	Diagnostic CT scan before treatment	19
	Diagnostic CT scan for follow-up	21
	MRI	12

**Table 2:** A summary of the anatomical distribution.

Anatomical sites	Quantity of patients (*n* = 19)	Quantity of lesions (*n* = 76)
Bone	14	34
Skull	11	21
Ribs	2	2
Sternum	1	1
Clavicle	1	1
Vertebra	5	5
Pelvis	3	3
Limbs	1	2
Lymph node	11	24
Neck	6	6
Clavicular region	3	3
Mediastinum	2	2
Abdomen	5	5
Retroperitoneal	4	4
Pelvic cavity	2	2
Inguinal region	1	2
Lung	3	5
Right lung	1	1
Both lungs	2	4
Liver	3	3
Spleen	3	3
Thyroid	1	1
Pituitary	1	1
Skin	1	1
Auricle	1	2
Labia	1	1

**Table 3:** The PET and diagnostic CT imaging profile.

Diagnostic profile	No. (%)
All FDG-avid lesions	69
FDG-avid lesions and abnormal on CT	59
FDG-avid lesions but normal on CT	15
Labia	1
Auricle	1
Spleen	3
Lymph node	4
Iliac	2
Vertebra	1
Femur	1
Humerus	1
Temporal	1
No FDG-avid lesions but abnormal on CT	5
Lung	2
Vertebral	1
Liver	1
Abdominal lymph node	1
No FDG-avid lesions and normal on CT	
Skin	1
Pituitary	1

**Table 4:** Classification and typing of the nineteen LCH patients.

Classification	Typing	Involved sites	No.
Single-system 6 cases	Single site 3 cases	Parietal bone	1
		Rib	1
		Frontal bone	1
	Multiple sites 3 cases	Skull + sternum + vertebral	1
		Skin	1
		Lung	1

Multisystem 13 cases	Low-risk group 1 case	Lymph nodes + thyroid gland + auricle + external labia	1
	High-risk group (invasion of liver, spleen, lung, and bone marrow) 12 cases	Bone marrow + lymph nodes	4
		Lymph nodes + spleen	1
		Bone marrow + lymph nodes + lung	1
		Lymph nodes + liver	1
		Bone marrow + lymph nodes + spleen	1
		Bone marrow + lymph nodes + lung + liver	1
		Bone marrow + lymph nodes + liver	1
		Bone marrow + spleen	1
		Bone marrow + pituitary	1

The article "Application of 18F-FDG PET/CT in Langerhans Cell Histiocytosis" was published in 2022. Journal: Contrast Media Mol Imaging.

## Data Availability

The datasets used and/or analyzed during the current study are available from the corresponding author on reasonable request.

## Abbreviations

LCH: Langerhans cell histiocytosis
CT: Computed tomography
PET: Positron emission tomography
AUC: Area under the curve
ROC: Receiver operating characteristic
EG: Eosinophilic granuloma.
